# Noninvasive bioluminescence imaging of the dynamics of sanguinarine induced apoptosis via activation of reactive oxygen species

**DOI:** 10.18632/oncotarget.7971

**Published:** 2016-03-08

**Authors:** Yan Wang, Beilei Zhang, Wei Liu, Yunpeng Dai, Yaru Shi, Qi Zeng, Fu Wang

**Affiliations:** ^1^ Engineering Research Center of Molecular and Neuro Imaging, Ministry of Education, School of Life Science and Technology, Xidian University, Xi'an, Shaanxi 710071, China; ^2^ Department of Gynecology and Obstetrics, Tangdu Hospital, The Fourth Military Medical University, Xi'an, Shaanxi 710038, China; ^3^ Department of Hepatobiliary Surgery, Xijing Hospital, The Fourth Military Medical University, Xi'an, Shaanxi 710032, China

**Keywords:** apoptosis, sanguinarine, luciferase reporter, bioluminescence imaging, therapeutic efficacy

## Abstract

Most chemotherapeutic drugs exert their anti-tumor effects primarily by triggering a final pathway leading to apoptosis. Noninvasive imaging of apoptotic events in preclinical models would greatly facilitate the development of apoptosis-inducing compounds and evaluation of their therapeutic efficacy. Here we employed a cyclic firefly luciferase (cFluc) reporter to screen potential pro-apoptotic compounds from a number of natural agents. We demonstrated that sanguinarine (SANG) could induce apoptosis in a dose- and time-dependent manner in UM-SCC-22B head and neck cancer cells. Moreover, SANG-induced apoptosis was associated with the generation of reactive oxygen species (ROS) and activation of c-Jun-N-terminal kinase (JNK) and nuclear factor-kappaB (NF-κB) signal pathways. After intravenous administration with SANG in 22B-cFluc xenograft models, a dramatic increase of luminescence signal can be detected as early as 48 h post-treatment, as revealed by longitudinal bioluminescence imaging *in vivo*. Remarkable apoptotic cells reflected from *ex vivo* TUNEL staining confirmed the imaging results. Importantly, SANG treatment caused distinct tumor growth retardation in mice compared with the vehicle-treated group. Taken together, our results showed that SANG is a candidate anti-tumor drug and noninvasive imaging of apoptosis using cFluc reporter could provide a valuable tool for drug development and therapeutic efficacy evaluation.

## INTRODUCTION

Apoptosis, or programmed cell death, is central to regulate normal cell growth and development in all multi-cellular organism [1, 2]. The dysregulation of apoptosis could ultimately result in a variety of disorders, including autoimmune diseases, neurodegenerative diseases and tumors [3, 4]. Thus, stimulating tumor cell apoptosis is a potential strategy for cancer drug discovery and anti-cancer therapy [5, 6]. In fact, a number of natural agents have been shown to exert their anti-tumor effects via a variety of apoptosis-inducing mechanisms in cancer cells [7–9]. Several conventional approaches, such as Annexin V [10, 11] or TdT-mediated dUTP nick end labeling (TUNEL) [12] assays, have been widely employed to detect apoptosis progress by taking advantage of the characteristic biochemical changes occurring in apoptosis. However, these methods usually require lysing or fixing of cells. Importantly, they have serious shortcomings in their inabilities to discriminate necrotic from apoptotic cells, resulting in the failure of truly reflecting the intrinsically complex apoptotic process [13–15]. Moreover, the internucleosomal fragmentation is not always associated with histologic evidence of apoptosis [16, 17]. Therefore, to overcome these limitations, noninvasively real-time monitoring apoptosis in living organisms would be a great advance for better understanding of apoptotic process, rapid screening of apoptosis-related drugs and early evaluation of drug therapeutic efficiency [18].

To date, various imaging probes have been developed to noninvasively monitor apoptosis using different modality imaging techniques, including optical imaging, radionuclide imaging, magnetic resonance imaging (MRI), and multiple-modality techniques [19–21]. Most of the apoptosis probes were based on a peptide sequence, DEVD (aspartic acid-glutamic acid-valine-aspartic acid), which can be specifically recognized and cleaved by the apoptotic effector caspase-3 [22–27]. Caspase-3, one of the intracellular cysteine proteases, has been identified as a pivotal mediator in the initiation and propagation of apoptosis [28, 29]. However, due to the low sensitivity, some of these probes are not well suitable for real-time visualization of caspase-3 activation and screening the candidate drugs for dysregulated apoptosis *in vivo*. Recently Kanno A *et al.* and our group have developed two novel apoptosis reporter probes, cyclic firefly luciferase (cFluc) [30, 31] and cyclic HSV1-TK (cTK) [32, 33], by fusing two fragments of DnaE inteins to neighboring ends of luciferase or TK connected with DEVD. Upon cells undergoing apoptosis stimulated by exogenous drugs, caspase-3 is activated and cleaves the genetically encoded cFluc or cTK, leading to the restoration of luciferase or thymidine kinase activity that can be detected in living organisms by bioluminescence imaging (BLI) or positron emission tomography (PET) imaging. The response of cFluc or cTK upon caspase-3 activation was extremely quick, suggesting a robust tool for screening candidate compounds and monitoring the dynamics of apoptotic process triggered by these compounds.

In this study, given the easier manipulation and low cost of BLI, we employed cFluc reporter probe to screen potential apoptosis-inducing compounds from a number of natural agents. We showed that sanguinarine (SANG), a benzophenanthridine alkaloid derived from the root of *Sanguinaria Canadensis*, could stimulate apoptosis via activating the production of reactive oxygen species (ROS) in head and neck tumor cells and animal models. To our best knowledge, it is the first study to noninvasively monitor SANG-induced apoptosis process *in vivo* with BLI techniques. Our data showed the potential of cFluc reporter probe as a valuable tool for high-throughput drug screening and anti-tumor therapeutic evaluation in preclinical models.

## RESULTS

### Validation of 22B-cFluc stable cell line and drug screening

Firstly we established a stable cell line, named 22B-cFluc, by genetically engineering the apoptosis reporter gene cFluc [30, 31] into the head and neck cancer cell line UM-SCC-22B. Upon cells undergoing apoptosis stimulated by extrinsic drugs, caspase-3 would specifically cleave the cyclic luciferase and result in the recovery of luciferase activity that can be detected in animals by BLI techniques (Figure 1). To validate the stable cell line, we treated 22B-cFluc cells with doxorubicin (DOX), an effective apoptosis inducer [34]. As expected, the DOX treated cells resulted in significant increase of luciferase signal compared with blank or DMSO treated groups, confirming that cFluc is an effective reporter for sensing cell apoptosis (Figure 2A).

**Figure 1:** Scheme of cFluc reporter for monitoring apoptosis The N-terminal and C-terminal of luciferase are linked with DEVD sequence, which is a substrate of caspase-3. Upon caspase-3 activation during apoptosis, the DEVD is cleaved and the cyclic luciferase restores its activity, which could be determined by *in vitro* luciferase assay or *in vivo* bioluminescence imaging.

**Figure 2:** Validation of cFluc reporter and drug screen **A.** 22B-cFluc cells were treated with DMSO or DOX. Twenty-four hours later, the cells were collected in triplicates and assayed for luciferase activity using a luminometer. **B.** 22B-cFluc cells were treated with DMSO or 14 different natural agents for 24 h in triplicates. The cells were then harvested for luciferase activity assay using a luminometer. Data are reported as mean ±SD of three independent experiments. **p<0.01, ***p<0.001 vs. DMSO control.

To identify natural agents that induce cell apoptosis, 22B-cFluc cells were treated with 14 different natural agents for 24 h, and the luciferase activities were then measured. As shown in Figure 2B, one of the drugs, SANG, induced the most fold increase of luciferase intensity compared with DMSO treated group, suggesting SANG has the potential to induce cell apoptosis.

### Effects of SANG on cell viability and apoptosis induction

To determine the effects of SANG on cell viability, 22B-cFluc cells were stimulated with different concentrations of SANG for 24 h, and then a CKK-8 assay was performed. As shown in Figure 3A, the treatment with SANG decreased the proliferation of 22B cells in a dose-dependent manner. Therefore, we carried out further experiments to investigate whether the inhibitory effect of SANG on cell viability was due to apoptosis. First, western blotting assay (Figure 3B) showed that SANG treatment activated the expression of caspase-3, which is believed to be a central effector for the initiation and propagation of apoptosis [35]. Second, flow cytometry analysis demonstrated that the percentage of Annexin V-positive cells increased according to the concentration increase of SANG used in cells (Figure 3C). Taken together, these data suggest that SANG induces apoptosis in 22B cancer cells.

**Figure 3:** Effects of SANG on cell viability and apoptosis **A.** 22B-cFluc cells were treated with different concentrations of SANG for 24 h. Then the cell viability was determined with a CKK-8 assay. **B.** 22B-cFluc cells were treated with 4 μM SANG for 24 h. Then the cells were harvested and the cellular proteins were detected by western blot assay with anti-caspase 3 antibody. Actin was used as an internal control. Quantification of the protein expression from three independent experiments was also shown. **C.** 22B-cFluc cells were treated with different concentrations of SANG for 24 h. Then the cells were stained with FITC-Annexin V and PI for flow cytometry analysis. The apoptotic cells were determined by the percentage of Annexin V (+)/PI (−) cells and the percentage of Annexin V (+)/PI (+) cells. Quantification of the flow cytometry from three independent experiments was also shown. Data are reported as mean ±SD of three independent experiments. *p<0.05, **p<0.01, ***p<0.001 vs. control.

### *In vitro* real-time monitoring SANG-induced apoptosis

To further explore the usefulness of cFluc reporter in detecting apoptosis induced by SANG, 22B-cFluc cells were treated with different amounts of SANG. As shown in Figure 4A, an increase in luciferase activity with increasing concentration of SANG was observed. Meanwhile, the cytosolic extracts of 22B-cFluc cells treated with different dose of SANG were measured to detect cellular caspase-3 activity using Ac-DEVD-pNA, which is a validated caspase-3 substrate [36]. It is observed that the absorbance at 450 nm increased in a dose-dependent manner, indicating increased caspase-3 activity stimulated by SANG (Figure 4B). In view of the positive correlation between luciferase intensity and caspase-3 activity, it is feasible to monitor and quantify the apoptosis process induced by SANG with cFluc reporter.

**Figure 4:** SANG induced apoptosis in a dose- and time-dependent manner **A.** 22B-cFluc cells were treated with different concentrations (0.5, 1, 2, 4 μM) of SANG. Twenty-four hours later, the cells were collected in triplicates and assayed for luciferase activity using a luminometer. **B.** The cells were treated the same as (A) and incubated with Ac-DEVD-pNA as substrate for caspase-3. Then the released fluorescence products were measured using a caspase-3 activity assay kit (Beyotime Biotechnology, China) according to the manufacturer's instructions. **C.** 22B-cFluc cells were treated with different concentrations (0.5, 2, 4 μM) of SANG for 4 h before washing the cells and changing the medium. At different time points after, the cells were collected in triplicates and assayed for luciferase activity. The average luciferase activity was plotted against with the time after treatment started. Data presented as mean ± SD for the three independent experiments. *p<0.05, **p<0.01, ***p<0.001 vs. control.

To further investigate the efficacy of cFluc reporter in monitoring apoptosis in real-time, 22B-cFluc cells were treated with different concentrations of SANG. After exposure to indicated concentration of SANG for 4 h, the cells were washed and replaced with serum-containing fresh medium for continuous culture. At different time points, the cells were collected and assayed for luciferase activity. As shown in Figure 4C, the luciferase signal from 0.5 μM SANG treated cells was consistently increased and then decreased at 40 h. In contrast, the signal from 2 μM SANG treated cells reached a peak at 30 h and then began to decrease at later time point. Compared to 0.5 or 2 μM SANG treated cells, the 4 μM SANG treated group showed consistent increase of luciferase intensity with time and reached the maximum at 24 h, then decreased afterwards. The different apoptosis kinetics induced by different concentration of SANG may be attributed to the fact that the cells are more sensitive to a higher concentration of SANG, resulting in achieving the peak of luciferase activity at an earlier time point.

### Generation of ROS is involved in SANG-induced apoptosis

It is suggested that the intracellular ROS generation may be correlated with mitochondrial dysfunction and apoptosis induction in various cell types [37]. To explore whether the SANG-induced apoptosis was associated with ROS, we therefore measured the intracellular ROS production with the DCFH-DA fluorescence dye. As shown in Figure 5A, the ROS production increased with the increased concentration of SANG used in 22B cells. However, prior treatment of the cells with a well-known ROS antioxidant, N-acetylcysteine (NAC), greatly blocked the generation of ROS in the 4 μM SANG treated 22B cells, and the blockage was time-dependent (Figure 5B).

**Figure 5:** ROS production was involved in SANG-induced apoptosis **A.** The cells were treated with different concentrations of SANG for 1 h, and then incubated with 10 mM DCFH-DA for 30 min. The ROS production in the cells was determined by measuring the OD values at excitation/emission wavelengths of 488/525 nm with a fluorescence spectrophotometer. **B.** The cells were treated with 4 μM SANG for 1 h, or they were pretreated with 20 mM NAC for 1 h and further co-incubated with 4 μM SANG for the indicated times. Then the ROS production was measured by the same method above. **C, D.** The 22B-cFluc cells were treated with 4 μM SANG for 24 h, or they were pretreated with different concentrations of NAC for 1 h and further co-incubated with 4 μM SANG for another 24 h. Then the cells were (C) harvested in triplicates and assayed for luciferase activity or (D) incubated with Ac-DEVD-pNA and assayed for caspase-3 activity. Data presented as mean ± SD for the three independent experiments. **p<0.01, ***p<0.001 vs. control.

To further investigate whether SANG-induced ROS generation was involved in apoptosis induction, the cells were pretreated with different dose of NAC and then co-incubated with SANG for further 24 h. As shown in Figure 5C, blocking the ROS production by NAC prevented the SANG-induced apoptosis, reflected by the dose-dependent decreased of luciferase activity. Furthermore, the inhibitory effect of NAC on the generation of ROS was correlated to a significant inhibition of caspase-3 activity (Figure 5D). Taken together, these data suggest that ROS production is involved in SANG-induced cell apoptosis.

### SANG-induced apoptosis is associated with the activation of JNK and NF-κB signal pathways

It is reported that the activation of cell signaling pathways, such as nuclear factor-kappaB (NF-κB), c-Jun-N-terminal kinase (JNK) or P38 mitogen-activated protein kinase (p38 MAPK), is involved in the regulation of cell growth and cell death [38, 39]. Thus, to examine whether these signal pathways were activated during SANG-induced apoptosis process, the cells were pretreated with BAY11-7082, SP600125 or SB203850, which are specific inhibitors of NF-κB, JNK or p38 MAPK signal pathways, respectively. The cells were then co-incubated with SANG for another 24 h. As shown in Figure 6A, the pretreatment with BAY11-7082 or SP600125 significantly attenuated the SANG-induced apoptosis, evidencing by the inhibition of luciferase activity. In contrast, SB203850 had little effect on the luciferase signal change comparing with the cells treated with SANG alone. These results indicated that NF-κB and JNK pathways were activated during the apoptosis induced by SANG.

**Figure 6:** SANG-induced apoptosis is associated with the activation of JNK and NF-κB **A.** The 22B-cFluc cells were treated with 4 μM SANG for 24 h, or they were pretreated with BAY11-7082, SP600125 or SB203850 for 1 h before co-incubating with SANG for 24 h. Then the cells were collected in triplicates for luciferase activity assay. **B.** The cells were treated with 4 μM SANG for 24 h and then harvested for western blot analysis of JNK p-JNK and IκBa protein expression using the indicated antibodies. Data presented as mean ± SD for the three independent experiments. **p<0.01, ***p<0.001 vs. control.

To further validate the involvement of NF-κB and JNK in SANG-induced apoptosis, the protein expression of IκBα and phosphorylated JNK (p-JNK) in cells treated with SANG were determined using western blotting assay. As shown in Figure 6B, stimulation of 22B cells with SANG resulted in the remarkably increased expression of p-JNK and IκBα, confirming that the activation of NF-κB and JNK was participated in SANG-mediated apoptosis in 22B cells.

### *In vivo* real-time imaging of SANG-induced apoptosis and therapeutic efficacy

To evaluate the apoptosis induced by SANG *in vivo*, 22B-cFluc cells were inoculated subcutaneously into one flank of nude mice and xenograft models were allowed to establish. Mice were treated intravenously with 10 mg/kg of SANG. At 24, 48 and 72 h after treatment, bioluminescent imaging was performed after i.p. injection of mice with 150 mg/kg of D-luciferin substrate. As shown in Figure 7A and 7B, SANG treatment induced an obvious increase of luminescent signal as early as 48 h after initial treatment. A sustained BLI intensity increased was observed throughout the course of experiment. At 72 h after treatment, the tumors were collected and subjected to TUNEL staining for evaluating apoptosis. Compared with the control tumors, the group treated with SANG exhibited significantly more cell apoptosis, indicated by the increased green signals from the sporadic apoptotic cells (Figure 7C).

**Figure 7:** *In vivo* real time imaging of SANG-induced apoptosis **A.** 22B-cFluc cells were implanted subcutaneously in nude mice (n=6). Three weeks later, mice were injected intravenously with 10 mg/kg of SANG. At the indicated time point after treatment, bioluminescent imaging (BLI) was performed after i.p. injection of mice with 150 mg/kg of luciferin. Representative BLI images were shown. **B.** The BLI signal from the region of interest in tumors was quantified. **C.** Representative images of TUNEL staining of tumor sections (20x magnification). Green color indicates positive apoptotic cells. Blue color indicates normal cell nuclei stained by DAPI.

To further explore the anti-tumor efficacy of SANG *in vivo*, the 22B-cFluc tumor bearing mice were treated intravenously with SANG at 10 mg/kg every other day throughout the experimental periods. As reflected by the tumor growth curve (Figure 8A), the treated mice showed response to SANG after 3 days and exhibited significant tumor growth retardation over time compared with control mice. After three weeks of treatment, the tumor burdens in SANG treated mice were reduced by 60% in comparison with that in control group, indicating the strong therapeutic efficacy of SANG. Note that there was a little body weight loss observed in both groups at the end of the experiment, which may be due to the toxicity of DMSO solvent towards the animals (Figure 8B). Taken together, these data confirm that SANG could efficiently induce apoptosis and tumor growth inhibition *in vivo*.

**Figure 8:** *In vivo* therapeutic efficacy evaluation of SANG 22B-cFluc cells were implanted subcutaneously in nude mice (n=6 each group). Three weeks later, mice were injected intravenously with 10 mg/kg of SANG or DMSO every other day throughout the experimental course. Then the **A.** tumor volumes and **B.** body weights of each mouse were recorded every 3 days for total of 21 days.

## DISCUSSION

It is believed that most chemotherapeutic agents inhibit tumor progression mainly by inducing a final pathway that leads to apoptosis, and resistance to anti-tumor treatment is widely thought to associate with deregulation of cell proliferation that enable apoptosis [40–42]. A few chemotherapeutic drugs, including doxorubicin and paclitaxel, are generally considered as active agents in a wide range of human tumors. However, the treatments are usually abeyant due to the drug resistance and intolerable toxicity [43, 44]. Therefore, there is a continuing need to explore novel anti-tumor drugs for overcoming these limitations. Natural products are an abundant source for cancer treatment. A large number of plant-derived drugs possess significant anticancer activities and have been increasingly used in cancer chemotherapy [45]. In the present study, we showed the utilization of cFluc reporter to screen pro-apoptotic natural compounds and to noninvasively monitor the dynamics of apoptotic process induced by a natural agent SANG in 22B head and neck tumor models. Our data demonstrated that SANG stimulated cell apoptosis in a dose- and time-dependent manner and the induction of apoptosis is involved in the generation of ROS as well as activation of JNK and NF-κB signal pathways.

The natural alkaloid SANG, derived from the root of *Sanguinaria Canadensis*, has been shown to exhibit potent anti-bacterial and anti-inflammatory activities as well as apoptosis-inducing activities in various cancer cells [46]. However, most of the results were concluded from *in vitro* cellular assays, which could not provide the kinetic patterns of apoptosis process induced by SANG. Molecular imaging enables noninvasively real-time visualization of cellular function and the subsequent molecular process in living subjects. Accordingly, noninvasive imaging of apoptosis would greatly aid in the verification of experimental therapeutics for drug screen and development [18]. Reporter genes have emerged as powerful imaging tools that can reflect the progression of a specific molecular event at the cellular level [47]. To date, several luciferase- or radionuclide-based reporter genes have been developed to visualize and quantify apoptosis in a noninvasive manner [22–25, 30, 32]. These reporter systems mainly concentrated on generating cells that stably expressing a modified reporter protein separated by a DEVD sequence, which is specifically cleaved by the caspase-3 protease. In these models, signal production occurs until the cells undergo apoptosis, at which time BLI or PET imaging could capture the signals. However, a drawback in these fusion protein reporters is the relatively large molecular size that would reduce the transfection or transduction efficiency into host cells [24, 25]. In addition, as is the case with those split luciferase reporters, the luminescence signal may be diminished due to the insufficient interaction between peptides that connecting with respective domain of luciferase [22, 23]. Comparing with these reporter probes, the cFluc or cTK reporters showed high sensitivity and free background noise during apoptosis [30, 32], which was also evidenced by our *in vitro* cellular results and *in vivo* imaging results in this study.

It is generally considered that apoptosis is a dynamic and complicated process and altered treatment even by the same drug in different tumor types may induce apoptosis that are associated with different signal pathways. Choi *et al*. [48] reported that the JNK pathway was activated in a ROS-dependent manner within half an hour of SANG treatment in human bladder cancer cells. However, a specific JNK inhibitor, SP600125, pretreatment did not attenuate the apoptosis induced by SANG, suggesting that ROS-dependent JNK activation cannot mediate the SANG-induced apoptosis in bladder caner cells. In another study [49], the same research group demonstrated that treatment of human colorectal cancer HCT-116 cells with SANG led to activation of p38MAPK and JNK pathways, but the disruption of these two pathways by specific inhibitors did not significantly prevent SANG-induced apoptosis in HCT-116 cells. In contrast, in the present study we found that the phosphorylation of JNK and increased expression of IκBα were detectable following SANG treatment in 22B human head and neck cancer cells. Furthermore, the pro-apoptotic effects induced by SANG was extremely blocked by the pretreatment with BAY11-7082 or SP610025 but not SB203850 inhibitor, suggesting that activation of NF-κB and JNK signal pathways were involved in SANG-inducing apoptosis in 22B cells. We speculate that the inconsistences among these reports are attributed to the different tumor types used.

With the cFluc reporter genetically modified human head and neck cancer cells, we successfully real-time assessed the dynamics of SANG-induced apoptosis in a noninvasive manner. Although the light absorption and scattering by mammalian tissues largely limit the usefulness of BLI techniques in deep tissues, it is indeed an ideal tool for high-throughput drug screening in preclinical setting. Firstly, BLI is relatively cost effective, simple and short acquisition time needed. Furthermore, BLI enables longitudinal monitoring of disease progression within the same animal, which would provide assistances to evaluate the optimal time intervals for imaging with other techniques including PET. It is noteworthy that although BLI have proved effective in preclinical trials, it is yet to be fully validated as useful tool in clinical applications. Radionuclide reporter probes such as cTK are more promising for visualizing apoptosis and drug response in a clinical setting [32, 33]. Our future work will proceed towards the clinical translation of the cTK probe for apoptosis-related drug development and therapeutic evaluation.

## MATERIALS AND METHODS

### Chemical drugs

The 14 natural drugs (Tubeimoside I, Betulinic acid, Ursolic acid, Neohesperidin, Sophocarpine, Diosmetin, Dioscin, Amygdalin, Oleanic acid, solanesol, Sparteine, Sanguinarine, Sclareolide, Harmine) and doxorubicin were purchased from Sigma. The signal pathway inhibitors BAY11-7082, LY294002 and SB203850 were purchased from Beyotime Biotechnology, China.

### Cell lines and transfection

The UM-SCC-22B cells were purchased from Cell Bank of Chinese Academy of Sciences (Shanghai, China) and maintained in DMEM medium, which supplemented with 10% fetal bovine serum (FBS), 1% glutamine, 100 mg/ml streptomycin and 100 U/ml penicillin (Invitrogen, CA). In order to establish the stable cell lines that express the cyclic firefly luciferase (cFluc), cFluc plasmid [30] was transfected into 22B cells with Lipofectamine 2000 (Invitrogen, CA) according to the manufacture's protocols. After 24 h, the cells were changed with selective medium containing 800 mg/mL G418 ((Invitrogen, CA)) every 3 days until clones were formatted. The cell clones were then picked up in 24-well plates and treated with doxorubicin. The luciferase activity of the clones was determined using luminometer (T20/20, Promega). The selective positive cell clone was identified and named as 22B-cFluc.

### Firefly luciferase assay

To validate the cyclic reporter, 22B-cFluc cells were seeded at a density of 3 × 10^5^/ml in a 24-well plate and treated with doxorubicin. 24 h later, D-luciferin was added in each well at a final concentration of 150 mg/ml, the cells were then lysed and the luciferase activity was measured using luminometer (T20/20, Promega). In the other experiments, the 22B-cFluc cells were treated with different concentration of SANG or 14 different types of drugs at the final concentration of 4 mM for each drug.

### Cell viability assay

The cell viability of SANG was determined by CCK-8 assay using a cell counting kit-8 (Beyotime Biotechnology, China) according to the manufacture's protocols. Briefly, cells were seeded in a 96-well plate (5 × 10^3^ cells/well) and treated with different concentrations of SANG (0.5 μM, 1 μMc, 2 μM, 4 μM) for 24 h. Then 10 ml CKK-8 was added to each well for 4 h and the absorbance at 450 nm was measured with a microplate reader (Synergy HT, Biotech). The optical density (OD) values were determined to reflect the viable cell populations from each well.

### Western bolt

The cells were harvested and were lysed in RIPA lysis buffer (Beyotime Biotechnology, China) at room temperature for 10 min. The supernatants were collected and the protein concentrations were determined using a BCA protein assay kit (Beyotime Biotechnology, China). Equal amounts of protein extracts (20 μg) were loaded in the SDS-PAGE gel and transferred to polyvinylidene difluoride (PVDF) membranes. After blocking with 5% nonfat dry milk for 1 h at room temperature, the transferred membranes were incubated with anti-caspase-3, anti-JNK, anti-p-JNK, anti-IκBα or anti-actin primary antibodies for 1 h at room temperature, then incubated with the IgG-HRP secondary antibody for another 1 h. The immunoreactivity was detected using ECL detecting instrument (GE Healthcare Bio-Sciences Corp). The primary and secondary antibodies were purchased from Santa Cruz Biotechnology Inc. (Santa Cruz, CA, USA). The protein bands were quantified using Image J software and normalized to the signal intensity of actin.

### Flow cytometry analysis

The apoptosis of cells induced by SANG was detected using an Annexin V-FITC/PI Apoptosis Detection Kit (BD Pharmingen, MI) according to the manufacturer's protocols. Briefly, the cells were harvested and washed twice with PBS. Then the cells were suspended in 1 ml annexin-V binding buffer, which contains 140 mM NaCl, 10 mM HEPES/NaOH and 2.5 mM CaCl_2_. The cells were incubated with Annexin V-FITC at room temperature for 15 min. PI (5 μg/ml) was added and the apoptotic cells were analyzed with a Accuri C6 flow cytometer (C6, BD Pharmingen, MI). The C Flow Plus software was used to determine the relative DNA content.

### *In vitro* caspase-3 activity assay

The caspase-3 activity was measured using a caspase-3 activity assay kit (Beyotime Biotechnology, China) according to the manufacturer's instructions. Briefly, the cells treated by different concentrations of SANG (0.5 μM, 1 μM, 2 μM, 4 μM) or control DMSO were collected, washed and lysed in a lysis buffer for 30 min on ice. The supernatants were then collected by centrifuging at 1,2000 rpm for 10 min. The Ac-DEVD-pNA (2 mM) was added to each sample and incubated at 37°C for 1 h. The optical density (OD) of each sample was finally quantified at a wavelength of 405 nm using a spectrophotometer (Shimadzu, Japan). The p-NA standard was used to calibrate the caspase-3 activity of each sample.

### ROS measurement

Intracellular ROS production was measured using a ROS assay kit (Beyotime Biotechnology, China) according to the manufacturer's instructions. Briefly, the cells were seeded at 24-well plates and treated by different concentrations of SANG or NAC for different periods of time. The cells were added with 10 mM DCFH-DA and incubated for 30 min at 37°C. The ROS production in the cells was determined by measuring the OD values at excitation/emission wavelengths of 488/525 nm using a fluorescence spectrophotometer (Shimadzu, Japan).

### *In vivo* animal studies

All animal experiments were performed in accordance with the Guild for the Care and Use of Laboratory Animals and with animal protocols approved by Xidian University. Xenografted tumor models were prepared by injection of 1×10^7^ 22B-cFluc cells suspended in PBS into nude mouse (n=6). After tumors reached a volume of approximately 100 mm^3^, SANG (10 mg/kg) was i.v. injected into mice. After injection for 24 h, 48 h and 72 h, mice were given a single i.p. dose of 150 mg/kg D-luciferin and bioluminescence imaging were performed using a Xenogen Lumina II system. The signal intensity in the region of interest was expressed as p/sec/cm2/sr using the Living Image software 4.1 (Xenogen). For the anti-tumor therapy studies, one group of tumor-bearing mice (n=6) received intravenously 10 mg/kg of SANG every other day throughout the experimental period, while the control group of mice (n=6) received DMSO only. Tumor growth measurement was calculated as *LW*^2^/2, where *L* indicates the long diameter and *W* indicates the short diameter.

### TUNEL staining

The mice were sacrificed and tumor samples were collected and sectioned. DNA fragments was determined by terminal deoxynucleotidyl transferase mediated dUTP nick end labeling (TUNEL) assay using a In situ Apoptosis Detection Kit (Merck Millipore) according to the manufacturer's protocols.

### Statistical analysis

Data are expressed as mean ± SD. Statistical comparisons were performed using software GraphPad Prism 5. Significant differences between the groups were determined using the unpaired Student's t-test. P value < 0.05 was accepted as an indication of statistical significance.

## CONCLUSIONS

In conclusion, the present study showed successful monitoring apoptotic events in response to a natural agent SANG via activation of ROS in head and neck tumor cells and xenografted tumors. Although there is still a long way to translate the unique caspase reporter cFluc into clinical settings, this molecular probe will provide a valuable tool for high-throughput screening of various pro-apoptotic or anti-apoptotic drugs and for monitoring their therapeutic efficacy.
